# Inguinal Hernia Containing an Inflamed Appendix: A Case of Amyand Hernia

This article has been retracted.

**DOI:** 10.7759/cureus.21121

**Published:** 2022-01-11

**Authors:** Deena M Aldosari, Nourh K Alaboon, Mohammed Y Mojammami, Mohammed O Aqeeli, Omar A Aldhafeeri, Ali A Theban, Ammar Y Bafarat, Najd A Almutairi, Mohammed H Alotaibi, Ali M Humood, Emad Y Alqurashi, Abdulmajed A Alramih, Abdulgader A Mira, Abdulhakeem M Khan, Faisal Al-Hawaj

**Affiliations:** 1 College of Medicine, King Saud University, Riyadh, SAU; 2 College of Medicine, Princess Nourah Bint Abdul Rahman University, Riyadh, SAU; 3 College of Medicine, Jazan University, Jazan, SAU; 4 College of Medicine, King Abdulaziz University, Jeddah, SAU; 5 College of Medicine, Shandong University, Jinan, CHN; 6 General Practice, Ministry of Health, Riyadh, SAU; 7 College of Medicine, King Saud Bin Abdulaziz University for Health Sciences, Jeddah, SAU; 8 College of Medicine, Imam Abdulrahman Bin Faisal University, Dammam, SAU; 9 College of Medicine, Arabian Gulf University, Manama, BHR; 10 College of Medicine, Taif University, Taif, SAU; 11 College of Medicine, Dar Al Uloom University, Riyadh, SAU; 12 College of Medicine, Marmara University, Istanbul, TUR

**Keywords:** inguinal hernia, acute appendicitis, scrotal swelling, appendix, amyand hernia

## Abstract

Inguinal hernia is a prevalent surgical condition worldwide. The hernia sac typically contains the omentum and small intestine. However, it has been reported that some other organs might be seen, including the ovary, fallopian tube, bladder, and colon. We report the case of a 23-year-old man who presented to our emergency department with the complaint of scrotal pain for the last six days. The pain was mainly in the right side. There was no history of preceding trauma, and the pain developed gradually. He described the pain as having a sharp nature and was constant. He reported having a low-grade fever that resolved with the use of over-the-counter analgesics. There was no change in the urine or bowel habits. No penile discharge was reported. On examination, the patient had a low-grade fever and tachycardia. The patient appeared in pain and was not cooperative to have a complete genitalia examination. However, there was a positive cough impulse in the right inguinal region. The laboratory findings suggested the presence of inflammatory or infectious processes with elevated leukocytes, C-reactive protein, and erythrocyte sedimentation rate. The patient was prepared for emergency laparotomy for reduction of the hernia and resection of the appendix. During exploration, the appendix was reduced from the hernia sac. The appendix appeared edematous, with marked erythema representing acute appendicitis. The appendix was resected and the hernia sac was closed. The presence of an appendix in the inguinal hernia sac is very rare. The preoperative diagnosis of Amyand hernia, the inguinal hernia containing the appendix, can be difficult based on the clinical presentation. Early diagnosis is crucial to avoid the potential complications of Amyand hernia, including perforation and abscess formation. Imaging studies can establish the diagnosis of Amyand hernia with high accuracy and confidence.

## Introduction

Inguinal hernia is one of the most common indications for abdominal surgeries worldwide. It is caused by a defect in the abdominal wall. The diagnosis of inguinal hernia is readily made by history taking and appropriate physical examination [1]. Imaging studies may be warranted in selected patients to diagnose occult hernias and to identify potential complications. Once diagnosed, symptomatic inguinal hernia must be surgically repaired promptly to avoid incarceration and strangulation [2]. In the majority of cases, the inguinal hernia sac contains only the omentum or the small intestine [1]. However, in unusual conditions, the inguinal hernia may contain the ovary, fallopian tube, colon, and urinary bladder. It is very rare to have the appendix in the hernia sac of inguinal hernia, which is termed the Amyand hernia. Here, we report the case of an inguinal hernia containing the appendix. The occurrence of inguinal hernia containing the appendix with the presence of acute appendicitis is rare.

## Case presentation

A 23-year-old man presented to our emergency department with the complaint of scrotal pain for the last six days. The pain was mainly in the right side. There was no history of preceding trauma, and the pain developed gradually. He described the pain as having a sharp nature and was constant. He reported having a low-grade fever that resolved with the use of over-the-counter analgesics. He did not identify any factors that aggravated or alleviated his pain. On the 10-point severity scale, he scored his pain as 5 in severity. No previous similar episodes of this pain were reported. There was no change in the urine or bowel habits. No penile discharge was reported.

The patient was otherwise healthy with no comorbidities and no previous abdominal surgeries. He underwent a tonsillectomy at the age of five years due to recurrence episodes of acute tonsillitis. The medication history included multivitamin tablets only. He smoked occasionally and had no history of alcohol consumption. He was a nursing student. The patient was single. He had no history of sexual activity or sexually transmitted diseases. The family history was positive for cystic fibrosis.

On examination, the patient had a low-grade fever of 38.0℃ and tachycardia with a pulse rate of 112 bpm with normal blood pressure (115/78 mmHg) and respiratory rate (14 bpm). The patient appeared in pain and was not cooperative to have a complete genitalia examination. However, there was a positive cough impulse in the right inguinal region. Abdominal examination revealed tenderness in the lower abdomen with no rigidity or guarding. Other systems had normal findings on physical examination.

The following laboratory findings suggested the presence of inflammatory or infectious processes: leukocytes (11,500/μL), C-reactive protein (17.2 mg/dL), and erythrocyte sedimentation rate (33 mm/hour). Other hematological and biochemical markers showed no derangement. The patient underwent computed tomography (CT) of the abdomen and pelvis, which demonstrated the right inguinal hernia containing the appendix that signs of inflammation, such as wall thickening and standing of the adjacent fat (Figures 1, 2).

**Figure 1:** Axial CT image showing the presence of right-sided inguinal hernia (arrow). CT, computed tomography

**Figure 2:** Coronal CT image showing the appendix (arrows) herniating to the right inguinal hernia. CT, computed tomography

The patient was prepared for emergency laparotomy for reduction of the hernia and resection of the appendix. During exploration, the appendix was reduced from the hernia sac. The appendix appeared edematous with marked erythema representing acute appendicitis. The inflamed appendix (Figure 3) was resected and the hernia sac was closed. A non-absorbable mesh was applied to repair the hernia defect. The operation was completed successfully with no complications. Histopathological examination of the appendix confirmed the presence of acute inflammation. The patient resumed oral feeding on the second postoperative day. He was discharged on the fourth postoperative day. He was followed up twice, after two weeks and then three months, and reported no active issues with no signs of recurrence.

**Figure 3:** Operative image showing the appendix with signs of acute inflammation.

## Discussion

We reported the case of acute appendicitis occurring in the setting of Amyand hernia. A hernia is defined as a protrusion of a viscus or its fascia through a defect in the containing cavity. Inguinal hernia classically contains the omentum. The presence of the appendix in the inguinal hernia sac is seen in less than 1% of all cases of inguinal hernia [1]. This surgical finding was first described by Claudius Amyand in 1735 in a young child with an inguinal hernia [3]. Furthermore, the occurrence of acute appendicitis in the setting of Amyand hernia is much rarer, with an incidence of less than 0.1% [4].

Previous studies indicated that Amyand hernia may have a mortality rate of up to 30% with a wound infection rate of 50% [2]. Much of this mortality rate is attributed to delayed diagnosis and the development of severe sepsis because of acute appendicitis. However, later studies showed that the rate of complications is much less common with a mortality rate of 5% only. This is related to the early diagnosis and management of Amyand hernia in the presence of imaging modalities and improved postoperative care [4]. In the present case, there was on delay in the diagnosis and management, and the patient did not develop any postoperative complications.

The diagnosis of Amyand hernia can be difficult because of the lack of specific clinical signs and symptoms. However, it is reported that frequent presentation includes the periumbilical pain that radiates to the right iliac fossa along with the presence of a right inguinal hernia [5]. In the present case, however, the patient did not report any history of abdominal pain related to the inguinal swelling. An abdominal CT scan, as in our case, can establish the diagnosis with high confidence. Several complications have been reported with Amyand hernia. The appendix may develop perforation and abscess formation. This may spread to the adjacent testicle and the spermatic cord and can result in necrotizing fasciitis on rare occasions [3]. The management can be performed by the conventional open repair, but recently the laparoscopic approach is more performed [5].

## Conclusions

The presence of appendicitis in the inguinal hernia sac is very rare. The preoperative diagnosis of Amyand hernia can be difficult based on the clinical presentation. Early diagnosis is crucial to avoid the potential complications of Amyand hernia, including perforation and abscess formation. Imaging studies can establish the diagnosis of Amyand hernia with high accuracy and confidence.
